The article "Overexpression of SEZ6L2 and Immune Infiltration in Cancer Based on Gene Image Diagnosis" was retracted in 2025. Reasons: compromised peer review; a compromised editor; unreliable results or conclusions; concerns about the results or conclusions.

# Overexpression of SEZ6L2 and Immune Infiltration in Cancer Based on Gene Image Diagnosis

**DOI:** 10.1111/srt.70096

**Published:** 2024-10-03

**Authors:** Liangfu Ding, Jilin Zeng, Junyong Zhao

**Affiliations:** ^1^ Department of General Surgery Chongming Branch of Shanghai Tenth People's Hospital Tongji University School of Medicine Shanghai China; ^2^ Department of Thyroid and Breast Division of General Surgery Shanghai Tenth People's Hospital Tongji University School of Medicine Shanghai China

**Keywords:** bioinformatics, biomarker, breast cancer, immune infiltration, optical image diagnosis, prognosis, SEZ6L2

## Abstract

**Background:**

With the rapid advancement of optical image diagnostic technology, researchers are delving into the potential applications in the field of cancer diagnosis and treatment. The exact link between the SEZ6L2 gene and cancer immune infiltration remains elusive.

**Materials and Methods:**

This study aims to investigate the relationship between SEZ6L2 gene overexpression and cancer immune infiltration using optical image diagnostic technology, thereby presenting novel insights for enhancing cancer diagnosis and treatment strategies. Tissue samples obtained from cancer patients were meticulously analyzed to quantitatively assess the expression of the SEZ6L2 gene through light image diagnostic technology. Additionally, immunohistochemical techniques were employed to assess the nature and quantity of immune infiltrating cells within the cancerous tissues.

**Results:**

The enrichment pathways were found to include complement activation, circulating immunoglobulin mediated humoral immune response, protein activation cascade, immunoglobulin complex, and immunoglobulin. In addition, the expression of SEZ6L2 is closely related to the infiltration level of tumor infiltrating immune cells (TIICs), and there is a potential relationship between the expression of SEZ6L2 and different marker genes of TIIC.

**Conclusion:**

Increased SEZ6L2 mRNA expression in breast invasive carcinoma was significantly associated with negative prognosis and immune invasion. SEZ6L2 may be a novel prognostic biomarker and a potential immunotherapeutic target in BRCA.

## 1 Introduction

Breast cancer is the most commonly diagnosed cancer in women, and the leading cause of a high proportion of deaths [1]. Female breast cancer has overstepped lung cancer with an estimated 2.3 million new cases [2, 3]. At present, the treatment for BRCA mainly includes surgery, chemotherapy, endocrine therapy, and so on. Despite treatment, the 5‐year survival rate in breast cancer with metastasis remains poor. A total of 20%−30% of early breast cancer patients still die of metastatic disease [4]. This suggests that the current staging system is not enough to exactly forecast prognosis, nor represent the intra‐tumor heterogeneity of BRCA patients. Thus, it is imperative to improve the present diagnostic and therapeutic methods. Searching for new molecular targets to slow or halt disease progression is an urgent priority.

The article "Overexpression of SEZ6L2 and Immune Infiltration in Cancer Based on Gene Image Diagnosis" was retracted in 2025. Reasons: compromised peer review; a compromised editor; unreliable results or conclusions; concerns about the results or conclusions.

Many studies have indeed found that the microenvironment regulates breast cancer growth and metastasis, includes stromal cells and distinct immune cell subsets [5]. It has been widely appreciated that the constitution of cells in the tumor microenvironment (TME) plays a supervisory role in not only dynamically regulating cancer progression but also influencing therapeutic outcomes [6, 7]. The character and spread of the immune cell subtypes are revealed to promote a better understanding of their role in breast cancer prevention and treatment. Since the investigation of diverse marker genes for TIICs or potential immune mechanisms is essential [8].

Seizure Related 6 Homolog Like 2 (SEZ6L2) is a gene localized on the cell surface, which encodes a seizure‐associated protein and regulates a variety of biological functions. SEZ6L2 has been revealed to have implications in neuronal and particularly motor function development [9]. In oncology, up‐regulated SEZ6L2 serves as a negative prognostic marker in various tumor entities [10]. Similarly, SEZ6L2 has been found to expedite the proliferation and metastasis of breast cancer [11]. However, the clinical values and certain correlations with the immune microenvironment of SEZ6L2 in breast cancer are still not fully unconfirmed. The potential effects of SEZ6L2 in BRCA and the relationship between SEZ6L2 and TIICs remain uncertain.

Optical image diagnosis technology is widely used in the medical field, especially in cancer diagnosis shows great potential. Through optical imaging methods, high‐resolution imaging of tissue and cell structures can be achieved, providing doctors with a wealth of information to aid diagnosis. In recent years, with the continuous innovation and improvement of optical microscopy, optical coherence tomography (OCT), and other technologies, optical image diagnosis technology has become one of the important auxiliary means for early cancer screening and pathological diagnosis. In view of the relationship between SEZ6L2 gene overexpression and cancer immune infiltration, light image diagnostic technology has a unique advantage. The imaging technology based on the optical principle enables accurate observation and quantitative analysis of SEZ6L2 gene overexpression regions and immune cell infiltration. Optical image diagnosis technology can obtain high‐quality images of tissues and cells in real‐time. Combined with computer‐aided analysis technology, it can quickly and accurately identify and locate the overexpression region of the SEZ6L2 gene, and further analyze the spatial relationship and quantity ratio between the SEZ6L2 gene and immune cells, which provides a powerful tool for the study of cancer immune infiltration.

The article "Overexpression of SEZ6L2 and Immune Infiltration in Cancer Based on Gene Image Diagnosis" was retracted in 2025. Reasons: compromised peer review; a compromised editor; unreliable results or conclusions; concerns about the results or conclusions.

The immune system acts as a principal determinant role in tumor growth. The prognostic value of immune‐infiltration and the success of immunotherapy were completely demonstrated [12]. A large number of bioinformatic tools are now available to identify specific patterns of infiltrating immune cells. In this manuscript, we observed that increased expression of SEZ6L2 is correlated with negative clinical characteristics and risk factors for OS. We aimed to explore the potential correlation between tumor immunity and the expression of the SEZ6L2 using bioinformatic tools, which may guide clinicians to refine treatment and promote the survival of BRCA patients. Therefore, the study on the association between SEZ6L2 gene overexpression and cancer immune infiltration based on optical image diagnostic technology can not only expand the application field of optical imaging in cancer research, but also contribute to the in‐depth understanding of this association mechanism, and provide a new perspective and guidance for cancer diagnosis, treatment, and prognosis assessment.

## 2 Materials and Methods

### 2.1 TCGA Datasets

Genomics data from the TCGA platform contains the comprehensive molecular characterization of multiple cancer types [13]. We downloaded the transcriptional expression data of SEZ6L2 and explored clinical information such as stage, grade, age, pathology type, and survival time from the TCGA official website. Finally, the 18 chosen cancer types contained at least five samples in the adjacent normal group. Using TCGA level 3 HTSeq‐FPKM format data were standardized as transcripts per million reads (TPM) for further study. In the aspect of optical image diagnosis, these rich TCGA data are used as the basis, combined with advanced optical imaging technology. Real‐time high‐resolution imaging of cancer tissue samples accurately captures the cell structure and infiltration of immune cells in areas overexpressed by the SEZ6L2 gene. The advantage of optical imaging diagnostic technology is that it can provide intuitive and clear histological information, and combined with the association analysis of gene expression data, it is expected to reveal the relationship between the overexpression of SEZ6L2 gene and immune cell infiltration in different cancer types.

The article "Overexpression of SEZ6L2 and Immune Infiltration in Cancer Based on Gene Image Diagnosis" was retracted in 2025. Reasons: compromised peer review; a compromised editor; unreliable results or conclusions; concerns about the results or conclusions.

### 2.2 UALCAN Analysis

UALCAN is an interactive web portal to carry out specific TCGA gene expression data through in‐depth analyses [14]. The samples enrolled contained SEZ6L2 gene expression data and relevant clinical information, including TNM stage, age, ER, PR, Her2 status, and PAM50. In our research, UALCAN was chosen to investigate the comparison of the SEZ6L2 transcription level between breast invasive carcinoma tissues and normal samples, simultaneously among disparate sub‐types and sub‐stages. Our databases included all available breast cases on UALCAN. The mRNA expression data were characterized by mean ± SD.

### 2.3 Human Protein Atlas (HPA) Database Analyses

Human protein atlas (HPA) contains normal tissues and tumor tissues information regarding the expression profiles of human genes on the protein level [15]. In our study, the different expressions in SEZ6L2 protein levels between breast invasive carcinoma tissue and normal tissues were compared by using the HPA website.

### 2.4 Survival Analysis

The prognostic values of SEZ6L2 at the mRNA level were investigated in breast invasive carcinoma. ROC curve was applied to detect the cutoff value of SEZ6L2 [16]. Kaplan–Meier Plotter is a survival analysis tool customized for prognostic indications. The Kaplan–Meier method and multivariate Cox regression analyses were applied to evaluate the influence of various prognostic factors on the overall survival (OS) and progress free interval (PFI) of BRCA patients.

### 2.5 Optical Image Diagnosis

In order to achieve the light image diagnostic step, it is first necessary to obtain light images of breast invasive cancer tissue, which can be achieved by using high‐resolution imaging techniques such as devices such as digital pathology scanners or microscopes that provide high‐quality light images to capture subtle changes in cell and tissue structure.

After obtaining the light image, it is necessary to process and analyze the image, which is realized by using computer vision and image processing algorithms. Image processing techniques are used to enhance images to improve clarity and contrast. Then a segmentation algorithm is applied to separate the tissue region in the image from the background region in order to better analyze the characteristics and structure of the cells. The expression region of the SEZ6L2 gene is then labeled using specific immunostaining techniques, which can be achieved by using techniques such as immunohistochemical staining or immunofluorescence staining. Staining will cause the SEZ6L2 gene expression region to show a distinct color or fluorescence signal on the light image, thus facilitating its accurate capture and analysis.

The article "Overexpression of SEZ6L2 and Immune Infiltration in Cancer Based on Gene Image Diagnosis" was retracted in 2025. Reasons: compromised peer review; a compromised editor; unreliable results or conclusions; concerns about the results or conclusions.

By combining gene expression data and light image diagnostic techniques, regions of SEZ6L2 gene overexpression in breast cancer tissues can be visually observed, and cell features associated with SEZ6L2 expression can be simultaneously analyzed. The infiltration of immune cells in breast cancer tissues can also be observed by light image diagnosis. Through the comprehensive analysis of these data, we can reveal the biological characteristics of the SEZ6L2 gene in breast cancer, and explore its association with immune cell infiltration, so as to provide more accurate guidance for the diagnosis and treatment of breast cancer.

### 2.6 Differentially Expressed Gene (DEG) Analysis

According to the median score of SEZ6L2 expression, breast invasive carcinoma patients in TCGA were separated into high‐ and low‐SEZ6L2 expression groups. DEGs were screened out between two groups with the searching criterion FDR < 0.05 and |logFC|>1 [17]. The retrieved DEGs were visualized using a heatmap via R‐package. The relationship between the top 10 DEGs and SEZ6L2 was assessed through Spearman's correlation analysis.

### 2.7 Functional Enrichment Analysis

Functional enrichment analyses are a common technique focusing on specific oncogenic pathways, containing Gene Ontology (GO) and Kyoto Encyclopedia of Genes and Genomes (KEGG) analysis, which were implemented for the DEGs using the R package GOplot [18]. Gene set enrichment analysis (GSEA) was performed through the R package clusterProfiler [19, 20]. Adjusted *p* value <0.05 and false discovery rate (FDR) <0.25 were regarded as statistically significantly enriched function or pathway terms.

### 2.8 Protein‐Protein Interaction (PPI) Network Analysis

The Search Tool for the Retrieval of Interacting Genes (STRING) is an online database for the retrieval of interacting genes [21]. In our research, STRING was implemented to retrieve co‐expression genes and establish PPI networks with an interaction score >0.4. The correlation analyses between the SEZ6L2 and co‐expressed genes of breast invasive carcinoma were measured.

### 2.9 Tumor Immunity Estimation Resource (TIMER) Database Analysis

TIMER is an online web‐integrated repository portal for the analysis of tumor‐immune interactions, including a million samples of 32 types of cancer [22]. TIMER uses a deconvolution algorithm to deduce the abundance of TIICs from gene expression profiles [23]. We performed TIMER to explicate the relevance between the copy number variation (CNV) of SEZ6L2 and the abundance of six types of tumor‐infiltrating immune cells (TIICs: including CD4+ T cells, CD8+ T cells, B cells, neutrophils, macrophages, and dendritic cells). Subsequently, a correlation module draws the expression scatterplots to assess the relationship between SEZ6L2 and TIICs marker genes.

The article "Overexpression of SEZ6L2 and Immune Infiltration in Cancer Based on Gene Image Diagnosis" was retracted in 2025. Reasons: compromised peer review; a compromised editor; unreliable results or conclusions; concerns about the results or conclusions.

### 2.10 Tumor‐Immune System Interaction Database (TISIDB)

TISIDB is recognized as a comprehensive online resource for tumor immune system interaction [24]. In this manuscript, TISIDB was conducted to investigate SEZ6L2 expression and tumor‐infiltrating lymphocytes (TILs) in Pan‐Cancer. The involved abundance of TILs was deduced by gene set variation analysis based on the gene expression profile. The correlations between SEZ6L2 and TILs were in‐depth analyzed by Spearman's test.

All statistical analyses were performed with the Bioinformatics Online Database, R (version 3.6.3), and R package ggplot2 was used to visualize expression differences. A paired *t*‐test and Mann–Whitney U‐test were used to determine the differences between breast invasive carcinoma tissues and adjacent normal tissues. Kaplan–Meier and log‐rank tests were conducted with the survminer package (0.4.9) to evaluate the influence of SEZ6L2 on survival.

## 3 Results

### 3.1 Expression Level of SEZ6L2 and Relationships With Clinical Pathological Characteristics of BCRA Patients

To evaluate the SEZ6L2 mRNA expression pattern, we excluded 15 cancer types, which contained less than five samples in the adjacent normal group. According to the working data refers to 18 cancer types. The mRNA expression of SEZ6L2 was significantly overexpressed in 15 of all 18 cancer types compared with normal tissues (Figure 1A). It suggested SEZ6L2 was abnormally expressed across various cancer types. Figure 1 shows the expression pattern of SEZ6L2.

**FIGURE 1:** The expression pattern of SEZ6L2. (A) The mRNA expression of SEZ6L2 from Pan‐cancer perspective. (B) The mRNA expression levels of SEZ6L2 in 112 BRCA and matched‐adjacent normal samples. (C) The mRNA expression levels of SEZ6L2 in 1099 BRCA samples and 292 normal samples. (D) The protein levels of SEZ6L2 are based on HPA. Normal tissue, https://www.proteinatlas.org/ENSG00000174938‐SEZ6L2/tissue/breast#img. (E) The protein levels of SEZ6L2 are based on HPA. Tumor tissue, https://www.proteinatlas.org/ENSG00000174938‐SEZ6L2/pathology/breast+cancer#img. (ns, *p* ≥ 0.05; *, *p* < 0.05; **, *p* < 0.01; ***, *p* < 0.001).

To determine the discrepancy in SEZ6L2 mRNA and protein expression level in breast invasive carcinoma, we analyzed the data from TCGA and HPA datasets. As exhibited in Figure 1B, paired data analysis showed that the mRNA expression levels of SEZ6L2 in breast invasive carcinoma tissues (*n* = 112) were dramatically higher than in normal tissues (*n* = 112) (Figure 1B, 5.534 ± 1.406 vs. 4.218 ± 1.448, *p* < 0.001). Similarly, unpaired data analyses showed the same result, that the mRNA expression levels of SEZ6L2 in breast invasive carcinoma tissues (*n* = 1099) were significantly higher than normal tissues (*n* = 292) (Figure 1C, 4.617 ± 1.607 vs. 2.669 ± 1.270, Wilcoxon rank sum test, *p* < 0.001). Consistently, immunohistochemical data from the HPA database exhibited that the SEZ6L2 protein level in BCRA tissue was up‐regulated as well (Figure 1D,E).

The article "Overexpression of SEZ6L2 and Immune Infiltration in Cancer Based on Gene Image Diagnosis" was retracted in 2025. Reasons: compromised peer review; a compromised editor; unreliable results or conclusions; concerns about the results or conclusions.

Meanwhile, the sub‐group analysis of various pathologic characteristics in BRCA samples was implemented through UALCAN analysis. The sub‐group analysis on disease stage, ER, PR, Her2 status, and age showed that the expression of SEZ6L2 in BRCA patients was significantly higher than in the control group (2A‐2I). Logistic regression analysis results revealed that SEZ6L2 expression in ≤60 years was lower than >60 years (*p* < 0.001), that ER, PR Negative was lower than ER, PR Positive (*p *< 0.01), and that Her2 Negative was higher than Her2 Positive (*p* < 0.001). In addition to that, SEZ6L2 expression had nothing to do with the pathologic stage (Table 1).

**TABLE 1:** Clinicopathological characteristics of high‐ and low‐SEZ6L2 expression groups.

Characteristic	Total	Low expression of SEZ6L2	High expression of SEZ6L2	*p*
*n*	1083	541	542	
T stage, *n* (%)				0.631
T1	277 (25.6%)	146 (13.5%)	131 (12.1%)	
T2	629 (58.1%)	309 (28.6%)	320 (29.6%)	
T3	139 (12.8%)	70 (6.5%)	69 (6.4%)	
T4	35 (3.2%)	15 (1.4%)	20 (1.9%)	
N stage, *n* (%)				0.497
N0	514 (47.5%)	262 (24.6%)	252 (23.7%)	
N1	158 (14.6%)	179 (16.8%)	179 (16.8%)	
N2	116 (10.7%)	61 (5.7%)	55 (5.2%)	
N3	76 (7%)	32 (3%)	44 (4.1%)	
M stage, *n* (%)				0.768
M0	902 (83.3%)	459 (49.8%)	443 (48%)	
M1	20 (1.8%)	9 (1%)	11 (1.2%)	
Pathologic stage, *n* (%)				0.973
Stage I	181 (16.7%)	91 (8.6%)	90 (8.5%)	
Stage II	619 (57.2%)	310 (29.2%)	309 (29.2%)	
Stage III	242 (22.3%)	121 (11.4%)	121 (11.4%)	
Stage IV	18 (1.7%)	8 (0.8%)	10 (0.9%)	
Age, *n* (%)				0.002**
≤60	601 (55.5%)	326 (30.1%)	275 (25.4%)	
>60	482 (44.5%)	215 (19.9%)	267 (24.7%)	
Histological type, *n* (%)				0.717
Infiltrating Ductal Carcinoma	762 (70.4%)	405 (41.5%)	367 (37.6%)	
Infiltrating Lobular Carcinoma	205 (18.9%)	104 (10.6%)	101 (10.3%)	
PR status, *n* (%)				0.007
Negative	342 (31.6%)	193 (18.7%)	149 (14.4%)	
Positive	688 (63.5%)	322 (31.1%)	366 (35.4%)	
ER status, *n* (%)				<0.001***
Negative	240 (22.2%)	146 (14.1%)	94 (9.1%)	
Positive	793 (73.2%)	369 (35.7%)	424 (41%)	
HER2 status, *n* (%)				0.010**
Negative	558 (51.5%)	267 (36.7%)	291 (40%)	
Positive	157 (14.5%)	95 (13.1%)	62 (8.5%)	
PAM50, *n* (%)				<0.001
Normal	40 (3.7%)	26 (2.4%)	14 (1.3%)	
LumA	562 (51.9%)	240 (22.2%)	322 (29.7%)	
LumB	204 (18.8%)	106 (9.8%)	98 (9%)	
Her2	82 (7.6%)	51 (4.7%)	31 (2.9%)	
Basal	195 (18%)	118 (10.9%)	77 (7.1%)	

The article "Overexpression of SEZ6L2 and Immune Infiltration in Cancer Based on Gene Image Diagnosis" was retracted in 2025. Reasons: compromised peer review; a compromised editor; unreliable results or conclusions; concerns about the results or conclusions.

### 3.2 Prognostic Value of SEZ6L2 in BCRA

The value for SEZ6L2 was explored to distinguish breast invasive carcinoma samples from normal samples by ROC curve analysis. The ROC curve analysis indicated SEZ6L2 had an AUC value of 0.714 (95% CI: 0.677−0.750) (2J). At a cutoff of 5.756, SEZ6L2 had a sensitivity of 90.3% and a specificity of 48.4%. The negative predictive value was 98% and the positive predictive value was 15.1%. In this study, the relationship between SEZ6L2 expression and BRCA patients’ prognosis was determined through the Kaplan–Meier method. Figure 2A–J shows SEZ6L2 expression in the subgroup and survival analysis for SEZ6L2. The median value of SEZ6L2 expression was used as a cut‐off score, and the patients were separated into high and low SEZ6L2 expression groups. The results demonstrated that the OS and PFI of BRCA patients in the low SEZ6L2 expression group was significantly longer than the high SEZ6L2 expression group. (OS: 215.2 vs. 122.3 months, hazard ratio (HR) = 1.49, 95% CI = 1.06−2.08, *p* < 0.05; PFI: NA vs. 148.5 months, HR = 1.41, 95% CI = 1.01−1.98, *p* < 0.05) (Figure 2K,L).

**FIGURE 2:** SEZ6L2 expression in subgroup and survival analysis for SEZ6L2. (A–C) Box‐plot showing the relative mRNA expression of SEZ6L2 in different TNM stage BRCA samples. (D–F) Exhibiting the relative mRNA expression of SEZ6L2 in different ER, PR, and Her2 status. (G) Showing the relative mRNA expression of SEZ6L2 in normal subjects or patients with stage 1, 2, 3, or 4 BRCA. (H) Showing the relative mRNA expression of SEZ6L2 in different PAM50 status. (I) Box‐plot showing the relative mRNA expression of SEZ6L2 in BRCA patients aged ≤60 and >60 years. (J) ROC curve showed that SEZ6L2 had an AUC value of 0.714 to discriminate BRCA tissues from healthy controls. (K) Kaplan–Meier survival curves indicated that BRCA patients with high SEZ6L2 mRNA expression had a shorter OS than those with low‐level of SEZ6L2 (*p* = 0.021). (L) PFI for BRCA patients with high versus low SEZ6L2 (*p* = 0.046). (ns, *p* ≥ 0.05; *, *p* < 0.05; **, *p* < 0.01; ***, *p* < 0.001).

Subsequently, the association between the expression of SEZ6L2 and prognosis in different subgroups was computed. As shown in the forest plot (Figure 3), the outcomes of multivariate Cox regression analyses evaluated that SEZ6L2 expression (adjusted HR = 1.984, 95% CI = 1.206−3.263, *p* = 0.007), T4 stage (adjusted HR = 7.300, 95% CI = 2.583–20.633, *p* < 0.001), N3 stage (adjusted HR = 2.900, 95% CI = 1.060–7.933, *p* = 0.038), M stage (adjusted HR = 3.636, 95% CI = 1.426–9.272, *p* = 0.007), and age (adjusted HR = 2.916, 95% CI = 1.766–4.815, *p* < 0.001) were independent factors of OS in patients with breast invasive carcinoma. SEZ6L2 expression was significantly related to unfavorable prognosis and might be considered as a potential biomarker for predicting survival in BRCA patients. Figure 3 shows Forest map based on multivariate Cox proportional‐hazard regression analysis for OS.

The article "Overexpression of SEZ6L2 and Immune Infiltration in Cancer Based on Gene Image Diagnosis" was retracted in 2025. Reasons: compromised peer review; a compromised editor; unreliable results or conclusions; concerns about the results or conclusions.

**FIGURE 3:** Forest map based on multivariate Cox proportional‐hazard regression analysis for overall survival.

### 3.3 Screening of DEGs in BRCA

A total of 3914 genes were discrepantly retrieved between the groups with high and low expression levels of SEZ6L2, containing 276 upregulated DEGs (19.5%) and 3638 downregulated DEGs (80.5%) (adjusted *p* value <0.05, |Log2‐FC| > 1). The retrieved DEGs were visualized using a heatmap via R‐package (Figure 4A and Table 2). Immediately, the correlation between the top 10 DEGs (CARTPT, CHGB, CPLX2, CHGA, SYT4, AMER3, XKR7, CCDC92B, MUC2, and PCSK1) and SEZ6L2 are presented in Figure 4B.

**FIGURE 4:** SEZ6L2‐related DEGs and functional enrichment analysis. (A) Volcano plot of DEGs. (B) Heatmap of correlation between SEZ6L2 expression and the top 10 DEGs. (C) GO analysis of DEGs. (D) KEGG analysis of DEGs.

**TABLE 2:** Correlation analysis between SEZ6L2 and 28 types of TILs in BRCA.

TILs	rho	*p* value
Activated CD8 T cell (Act_CD8)	−0.165	3.60E‐08
Central memory CD8 T cell (Tcm_CD8)	−0.043	0.151
Effector memory CD8 T cell (Tem_CD8)	−0.247	1.14E‐16
Activated CD4 T cell (Act_CD4)	−0.303	2.20E‐16
Central memory CD4 T cell (Tcm_CD4)	−0.063	0.0369
Effector memory CD4 T cell (Tem_CD4)	−0.254	1.54E‐17
T follicular helper cell (Th)	−0.223	9.62E‐14
Gamma delta T cell (Tgd)	−0.169	1.67E‐08
Type 1 T helper cell (Th1)	−0.254	1.66E‐17
Type 17 T helper cell (Th17)	−0.14	3.01E‐06
Type 2 T helper cell (Th2)	−0.319	2.20E‐16
Regulatory T cell (Treg)	−0.178	3.16E‐09
Activated B cell (Act_B)	−0.235	3.65E‐15
Immature B cell (Imm_B)	−0.243	3.38E‐16
Memory B cell (Mem_B)	−0.338	2.20E‐16
Natural killer cell (NK)	−0.184	7.87E‐10
CD56bright natural killer cell (CD56bright)	−0.079	0.00895
CD56dim natural killer cell (CD56dim)	−0.014	0.654
Myeloid derived suppressor cell (MDSC)	−0.186	5.19E‐10
Natural killer T cell (NKT)	−0.239	1.17E‐15
Activated dendritic cell (Act_DC)	−0.107	0.000361
Plasmacytoid dendritic cell (pDC)	−0.001	0.98
Immature dendritic cell (iDC)	−0.071	0.0185
Macrophage (Macrophage)	−0.153	3.68E‐07
Eosinophil (Eosinophil)	−0.124	3.68E‐05
Mast cell (Mast)	−0.228	2.23E‐14
Monocyte (Monocyte)	−0.037	0.217
Neutrophil (Neutrophil)	0.017	0.568

### 3.4 Functional Enrichment Analysis

GO enrichment analysis indicated that DEGs were enriched in several different GO terms such as complement activation, humoral immune response mediated by circulating immunoglobulin, protein activation cascade, immunoglobulin complex, and immunoglobulin (Figure 4C and Table 3). In addition, other significantly DEGs‐enriched pathways included neuroactive ligand‐receptor interaction, taste transduction, alcoholism, nicotine addiction, and systemic lupus erythematosus were shown by KEGG pathway analysis (Figure 4D). Subsequently, GSEA was performed between the high‐ and low‐SEZ6L2 expression groups and more immune‐related biological processes were revealed to be significantly enriched in the low SEZ6L2 expression group, indicating that the high SEZ6L2 expression conferred a decreased immune phenotype in the breast invasive carcinoma (Figure 5A–D).

The article "Overexpression of SEZ6L2 and Immune Infiltration in Cancer Based on Gene Image Diagnosis" was retracted in 2025. Reasons: compromised peer review; a compromised editor; unreliable results or conclusions; concerns about the results or conclusions.

**TABLE 3:** Correlation analysis between SEZ6L2 and marker genes of immune cells in TIMER.

Description	Marker genes	None Cor	*p*	Purity Cor	*p*
CD8+ T cell	CD8A	−0.154	9.768E‐07	−0.138	1.267E‐05
	CD8B	−0.127	6.040E‐05	−0.106	8.035E‐04
T cell (general)	CD3D	−0.183	6.625E‐09	−0.172	4.495E‐08
	CD3E	−0.177	1.989E‐08	−0.166	1.411E‐07
	CD2	−0.189	1.774E‐09	−0.179	1.245E‐08
T cell exhaustion	PDCD1	−0.136	1.762E‐05	−0.116	2.385E‐04
	CTLA4	−0.212	1.476E‐11	−0.201	1.561E‐10
	LAG3	−0.133	2.395E‐05	−0.119	1.640E‐04
	HAVCR2	−0.150	1.914E‐06	−0.134	2.201E‐05
	GZMB	−0.216	6.108E‐12	−0.206	5.945E‐11
Th1	TBX21	−0.162	2.895E‐07	−0.147	3.385E‐06
	STAT4	−0.193	9.015E‐10	−0.183	5.778E‐09
	IFNG	−0.168	9.945E‐08	−0.153	1.287E‐06
	TNF	−0.105	8.610E‐04	−0.094	3.023E‐03
	STAT1	−0.095	2.780E‐03	−0.083	8.591E‐03
Th2	GATA3	0.186	3.172E‐09	0.174	3.207E‐08
	STAT5A	−0.066	3.679E‐02	−0.045	1.524E‐01
	STAT6	0.219	2.874E‐12	0.231	1.854E‐13
Tfh	BCL6	−0.035	2.687E‐01	−0.027	3.898E‐01
	IL21	−0.128	4.809E‐05	−0.115	2.879E‐04
Th17	STAT3	0.029	3.569E‐01	0.037	2.431E‐01
	IL17A	−0.053	9.319E‐02	−0.040	2.071E‐01
Treg	FOXP3	−0.173	4.208E‐08	−0.158	5.513E‐07
	CCR8	−0.167	1.209E‐07	−0.154	1.106E‐06
	TGFB1	0.069	3.006E‐02	0.107	7.119E‐04
	STAT5B	−0.020	5.348E‐01	−0.009	7.715E‐01
B cell	CD19	0.162	2.816E‐07	−0.146	3.716E‐06
	CD79A	−0.168	9.215E‐08	−0.154	1.064E‐06
	CD27	−0.161	3.371E‐07	−0.146	3.546E‐06
Natural killer cell	KIR2DL1	−0.111	4.313E‐04	−0.097	2.233E‐03
	KIR2DL3	−0.116	2.335E‐04	−0.101	1.379E‐03
	KIR2DL4	−0.172	4.661E‐08	−0.159	4.436E‐07
	KIR3DL1	−0.130	4.087E‐05	−0.114	3.045E‐04
	KIR3DL2	−0.170	6.359E‐08	−0.156	7.763E‐07
	KIR3DL3	−0.115	2.759E‐04	−0.105	8.727E‐04
	KIR2DS4	−0.120	1.507E‐04	−0.105	8.853E‐04
Monocyte	CD14	−0.041	2.017E‐01	−0.017	6.033E‐01
	CD86	−0.176	2.109E‐08	−0.162	2.757E‐07
	CSF1R	−0.045	1.515E‐01	−0.016	6.188E‐01
TAM	CD68	−0.128	5.209E‐05	−0.110	4.875E‐04
M1 macrophage	NOS2	0.038	2.334E‐01	0.042	1.844E‐01
	IRF5	0.006	8.416E‐01	0.023	4.746E‐01
	PTGS2	−0.121	1.235E‐04	−0.103	1.109E‐03
M2 macrophage	CD163	−0.115	2.815E‐04	−0.098	2.074E‐03
Neutrophil	CEACAM8	0.056	7.742E‐02	0.056	7.853E‐02
	ITGAM	−0.072	2.359E‐02	−0.051	1.082E‐01
	CCR7	−0.168	9.731E‐08	−0.154	1.060E‐06
Dendritic cell	CD1C	−0.083	9.078E‐03	−0.054	8.937E‐02
	NRP1	−0.064	4.268E‐02	−0.043	1.773E‐01
	ITGAX	−0.143	6.245E‐06	−0.125	7.828E‐05

The article "Overexpression of SEZ6L2 and Immune Infiltration in Cancer Based on Gene Image Diagnosis" was retracted in 2025. Reasons: compromised peer review; a compromised editor; unreliable results or conclusions; concerns about the results or conclusions.

**FIGURE 5:** GSEA of DEGs. (A) Hallmark gene sets deposited in MSigDB. (B) Biological processes of Gene Ontology gene sets downloaded from MSigDB. (C) Cellular compositions of Gene Ontology gene sets downloaded from MSigDB. (D) Molecular functions of Gene Ontology gene sets downloaded from MSigDB.

### 3.5 PPI Networks Analysis

Figure 6A exhibited the network of SEZ6L2 and its 10 co‐expression genes. The correlation between the expression of SEZ6L2 and co‐expressed genes (ASPHD1, CDIPT, HIRIP3, DOC2A, KIF22, PRRT2, and GRIA1RHOA) in breast invasive carcinoma from TCGA was demonstrated in Figure 6B–H.

**FIGURE 6:** PPI networks and correlation analyses. (A) A network of SEZ6L2 and its co‐expression genes. (B–H) The correlation analyses between the expression of SEZ6L2 and co‐expressed genes in BRCA.

### 3.6 Relationship Between SEZ6L2 Expression and Tumor‐Infiltrating Immune Cells

The TIMER database Analysis results demonstrated that the copy number variation (CNV) of SEZ6L2 was significantly related to the infiltration levels of CD8+ T cells, CD4+ T cells, B cells, macrophages, neutrophils, and dendritic cells (Figure 7A). Meanwhile, the distinction of 24 types of tumor‐infiltrating immune cells (TIICs) between the high‐ and low‐SEZ6L2 expression groups was compared. The results suggested that the low‐expression group had more activated T cells (*p* < 0.001), pDC (*p* < 0.05), NK CD56dim cells (*p* < 0.001), neutrophils (*p* < 0.01), macrophages (*p* < 0.001), iDC (*p* < 0.05), DC (*p* < 0.001), cytotoxic cells (*p* < 0.001), CD8 T cells (*p* < 0.001), B cells (*p* < 0.001), T helper cells (*p* < 0.001), Tcm (*p* < 0.05), Tem (*p* < 0.001), Th1 cells (*p* < 0.001), Th2 cells (*p* < 0.001) and TReg (*p* < 0.001), mast cell (*p* < 0.001), natural killer cell (*p* < 0.01), and monocyte (*p* < 0.05) infiltrates. The high‐expression group had more activated NK cells (*p* < 0.01), NK CD56bright cells (*p* < 0.001), and eosinophils (*p* < 0.01). Other TIICs showed no statistically significant intergroup differences (Figure 7B).

**FIGURE 7:** Relationship between SEZ6L2 expression and TIICs. (A) SEZ6L2 copy number variation affected the infiltration level of CD8+ T cells, CD4+ T cells, B cells, macrophages, neutrophils, and dendritic cells. (B) The distribution of 24 subtypes of immune cells in low and high SEZ6L2 expression groups. (ns, *p* ≥ 0.05; *, *p* < 0.05; **, *p* < 0.01; ***, *p* < 0.001).

The article "Overexpression of SEZ6L2 and Immune Infiltration in Cancer Based on Gene Image Diagnosis" was retracted in 2025. Reasons: compromised peer review; a compromised editor; unreliable results or conclusions; concerns about the results or conclusions.

In addition to that, Figure 8A showed the correlation between SEZ6L2 expression and 28 types of TILs across multiple cancer types. As shown in Figure 8B–L, the expression of SEZ6L2 was correlated with the abundance of Tem CD8 cell, Act CD4 T cell, Tem CD4 cell, Th, Th1, Th2, Act B cell, Imm B cell, Mem B cell, NKT, and Mast. These analysis reports indicated that SEZ6L2 may play a specific role in the immune microenvironment in breast invasive carcinoma. After adjustment of the purity, the correlation between SEZ6L2 and the diverse marker genes of TIICs was further investigated using the TIMER database.

**FIGURE 8:** Relations between SEZ6L2 expression and TILs. (A) Relations between SEZ6L2 expression and TILs across human cancers. (B–L) SEZ6L2 was correlated with abundance of Tem CD8 cell, Act CD4 T cell, Tem CD4 cell, Th, Th1, Th2, Act B cell, Imm B cell, Mem B cell, NKT, and Mast.

## 4 Discussion

The Sez6 family consists of Sez6, Sez6L, and Sez6L2, all three have been found to have an effect on synapse numbers and dendritic morphology. The five complement control protein (CCP) domains and 2−3 CUB domains are the common domains of Sez6 family, indicating that they may be involved in complement regulation [25]. Be short of Sez6 family proteins leads to phenotypes commonly associated with neuropsychiatric disorders [26]. SEZ6L2 is located in the region of chromosome 16p11.2 and has broad expression in the brain, stomach, and prostate glands, besides it is seldom in other normal tissues [27]. This gene is predicted to be relevant to autism spectrum disorders [28]. In oncology, upregulation of SEZ6L2 serves as a poor prognostic marker in several tumor entities, such as lung cancer, thyroid carcinoma, colorectal cancer, cholangiocarcinoma, hepatocellular Carcinoma, and ovarian cancer [29, 30, 31, 32, 33, 34]. In combination with light image diagnostic technology, high‐resolution imaging technology was used to accurately capture the overexpression region of SEZ6L2 gene in breast invasive carcinoma tissue. Through light image diagnosis, cell features related to SEZ6L2 expression in tissue structure and infiltration of immune cells can be visually observed. This research strategy combining gene expression data and light image diagnosis technology is expected to reveal the biological characteristics of SEZ6L2 gene in breast cancer and the association between SEZ6L2 gene and immune cell infiltration. In our study, we revealed the mRNA expression of SEZ6L2 is upregulated in breast invasive carcinoma tissues. On the basis of data, we also found that elevated expression of SEZ6L2 acts as an independent prognostic biomarker of poor OS and PFI in BRCA patients (*p* < 0.05).

The article "Overexpression of SEZ6L2 and Immune Infiltration in Cancer Based on Gene Image Diagnosis" was retracted in 2025. Reasons: compromised peer review; a compromised editor; unreliable results or conclusions; concerns about the results or conclusions.

In this manuscript, we summarized the relationships between SEZ6L2 expression and prognosis in different subgroups by multivariate Cox regression analyses. At the same time, we also confirmed that SEZ6L2 expression (adjusted HR = 1.984, 95% CI = 1.206−3.263, *p* = 0.007), T4 stage (adjusted HR = 7.300, 95% CI = 2.583–20.633, *p* < 0.001), N3 stage (adjusted HR = 2.900, 95% CI = 1.060–7.933, *p* = 0.038), M stage (adjusted HR = 3.636, 95% CI = 1.426–9.272, *p* = 0.007), and age (adjusted HR = 2.916, 95% CI = 1.766–4.815, *p* < 0.001) were independent factors of OS in patients with breast invasive carcinoma. Our research concluded that SEZ6L2 expression was significantly related to OS in BRCA patients and might be considered as a promising biomarker for predicting survival in patients with BRCA.

Currently, the function and mechanism of SEZ6L2 in tumors is still largely unclear. According to previous studies, SEZ6L2 has been indicated can be regulated by STAT3, which may elevate the expression of the vascular endothelial growth factor, promoting tumor angiogenesis and cancer progression [35, 36]. Investigations of the mechanisms indicated that knockdown SEZ6L2 expression impairs the growth of the colorectal cancer cells by inducing caspase‐dependent apoptosis [31]. Meanwhile, SEZ6L2 may upregulate the expression of PDGF, VEGF, and VEGF receptors through positive feedback regulation, thus ultimately promoting the angiogenesis of cholangiocarcinoma [32]. Other studies found SEZ6L2 plays a crucial part in oncogenic effects on breast cancer progression through multiple cancer‐related signaling pathways. Chen et al. identified a transcriptional factor called upstream transcription factor1 (USF1), which could promote SEZ6L2 expression to expedite the proliferation and metastasis of breast cancer [11]. All the current studies suggest that SEZ6L2 could be regarded as a novel biomarker or potential target for cancer therapy. Nevertheless, we need to warrant further exploration to investigate the biological function mechanism of SEZ6L2 in breast cancer.

In order to validate the clinical value of SEZ6L2 in BRCA, an ROC curve was applied. Our results show that SEZ6L2 had a significantly high AUC value in the detection of BRCA. We explored the DEGs correlated with SEZ6L2 and its co‐expression genes in BRCA tissues by GO, KEGG, GSEA enrichment analysis, and PPI networks. With the help of bioinformatic tools, we found that significantly enriched pathways included the complement activation, humoral immune response mediated by circulating immunoglobulin, protein activation cascade, immunoglobulin complex, and immunoglobulin were associated with high SEZ6L2 expression. Suggesting that the promoted expression of SEZ6L2 conferred a decreased immune phenotype in breast cancer. These findings require further experimental validation and may enrich the content of SEZ6L2‐related biological functions in BRCA.

The article "Overexpression of SEZ6L2 and Immune Infiltration in Cancer Based on Gene Image Diagnosis" was retracted in 2025. Reasons: compromised peer review; a compromised editor; unreliable results or conclusions; concerns about the results or conclusions.

A tumor is not a simple blend of cancer cells, but rather a heterogeneous collection of infiltrating and resident host cells, secreted factors, and extracellular matrix [37]. Tumors become infiltrated with diverse adaptive and innate immune cells that can perform both pro‐ and anti‐tumorigenic functions [38]. Additionally, Studies of both tumoral and systemic changes in the immune system following immune checkpoint inhibitors (ICI) therapy have yielded insight into the basis for both efficacy and resistance [39]. Up till now, the correlation between SEZ6L2 expression and immune cell infiltration in BRCA has not been investigated. In this manuscript, we disclosed that SEZ6L2 was significantly related to the infiltration levels of CD8+ T cells CD4+ T cells, B cells, macrophages, neutrophils, and dendritic cells. Meanwhile, we also found a correlation between SEZ6L2 expression and 28 types of TILs across human cancers. These data indicated that SEZ6L2 may play a specific role in immune infiltration in BRCA. Subsequently, the correlation between SEZ6L2 expression and the diverse marker genes of TIICs by the TIMER database was further investigated.

## 5 Conclusion

The study delved into the association between overexpression of SEZ6L2 in cancer and immune cell infiltration. Optical imaging diagnostic technology provides reliable and high‐resolution images of breast cancer tissue. Through the processing and analysis of these images, the overexpression region of the SEZ6L2 gene can be accurately captured and located, and the infiltration of immune cells in breast cancer tissues can be visually observed. Light image diagnosis provides visual indicators of breast cancer immune infiltration and provides a new way to better understand the immune environment and prognosis of breast cancer. The results showed that the expression level of SEZ6L2 was closely related to the degree of infiltration of various immune cell types, suggesting that SEZ6L2 plays an important role in regulating the tumor immune microenvironment. We demonstrated that SEZ6L2 was upregulated in BRCA patients. Increased expression of SEZ6L2 was correlated with clinical progression and regarded as a risk factor for survival. SEZ6L2 could be regarded as a potential prognostic indicator for BRCA patients. However, there are several limitations in this study. First, our data were gained from online public databases, so the sample contents maybe not impeccable, and we were not able to obtain all of the clinical information. Second, the impact of SEZ6L2 on immune infiltration in breast cancer needs further examination to detail the biological functions and the underlying mechanism.

The article "Overexpression of SEZ6L2 and Immune Infiltration in Cancer Based on Gene Image Diagnosis" was retracted in 2025. Reasons: compromised peer review; a compromised editor; unreliable results or conclusions; concerns about the results or conclusions.

## Conflicts of Interest

The authors declare no conflicts of interest.

## Ethics Statement

The authors have nothing to report.

## Data Availability

The data supporting the results of this study are available from the corresponding author.
